# An Information-Based Nursing Quality Evaluation Model of Daily PICC Work in Outpatient Clinics

**DOI:** 10.1155/2022/8187644

**Published:** 2022-07-21

**Authors:** Qingmei Yi, Xi Li, Tingting Chen, Zhiguo Li, Xiaohong Cao, Wei Gu

**Affiliations:** Hunan Children's Hospital, Changsha 410007, China

## Abstract

Our purpose of this study was to analyze the application value of the information-based nursing quality evaluation model in improving the daily work quality of the PICC room in the outpatient department. From January 2020 to December 2020, 465 patients who received PICC treatment were selected as the research objects and divided into the observation group (265 cases, July 2020–December 2020, information-based nursing quality evaluation model after implementation) and the control group (200 cases, January 2020–June 2020, before the implementation of the information-based nursing quality assessment model). Compared with the control group, the children and their families in the observation group had higher PICC health knowledge and compliance scores, longer mean time for catheter placement, lower overall complication rate, and higher overall satisfaction rate after the intervention. The information-based nursing quality evaluation model can improve the daily work quality of the PICC room in the outpatient clinic, improve the clinical efficacy of PICC in patients, and reduce the incidence of complications such as catheter shedding. It is worthy of clinical application.

## 1. Introduction

Peripherally inserted central venous catheters (PICC) are performed directly in the patient's peripheral vein (usually the upper arm vein), and the drug is infused directly into the patient's body through the intravenous line. This can effectively reduce the damage to the peripheral veins (arm veins) of the patient, reduce the stimulation of the blood vessels by the drugs, and reduce the chance of complications such as phlebitis [1, 2]. To further improve the quality of daily maintenance of PICC in outpatient clinics, this study proposes to adopt an information-based care quality assessment model to intervene in the care of PICC patients to ensure more effective protection of their peripheral vessels, reduce the incidence of complications such as catheter dislodgement, and improve their overall treatment efficacy. The study also investigates the practical application of this intervention model as follows.

## 2. Patients and Methods

### 2.1. Patients

From January 2020 to December 2020, 465 patients admitted to receive PICC treatment were selected as the study subjects and divided into the observation group (265 cases, from July 2020 to December 2020, after the implementation of the information-based nursing care quality assessment model) and the control group (200 cases, from January 2020 to June 2020, before the implementation of the information-based nursing care quality assessment model). Statistical analysis of the basic data of the two groups, such as age and gender composition, showed no statistical difference (*P* > 0.05), as shown in Table 1. The study was approved by the Ethics Committee of Hunan Children's Hospital.

The inclusion criteria were as follows: (1) all subjects in this study met the relevant clinical criteria by referring to the PICC Placement and Maintenance Manual [3]; (2) all patients and their families selected for the study voluntarily signed their consent and were approved by the Medical Ethics Committee. The exclusion criteria are as follows: (1) the child has severe coagulation disorders; (2) the child had developed complications such as infections; (3) the child had severe allergic reactions to medication or medical devices used; (4) the child had a history of phlebitis or venous thrombosis; (5) the child had a mental illness or cognitive impairment that prevents him/her from cooperating effectively with health care professionals in the treatment and intervention.

### 2.2. Intervention Methods

In the control group, from January 2020 to June 2020, i.e., before the implementation of the information-based quality of care assessment model, routine PICC placement maintenance was implemented, i.e., the child was registered in the outpatient clinic for intravenous therapy, a basic assessment of the child's PICC localization was performed by the outpatient specialist, maintenance items were prescribed according to the presence of complications and maintenance needs, and PICC placement maintenance was formally started. The intervention care of the observation group from July 2020 to December 2020, i.e., after the implementation of the information-based quality of care assessment model, was carried out in the following manner.

We first set up a professional informatics nursing quality assessment team: the nursing staff of the PICC unit in the outpatient clinic worked together to form an informatics nursing quality assessment team. The members of the team reviewed a large number of cases and literature, summarized and assessed the relevant nursing conditions during the maintenance of the previous PICC catheter placement, thoroughly explored and analyzed the main factors causing complications such as catheter dislodgement, and proposed corresponding nursing care interventions based on the relevant factors. The interventions were based on these factors. At the same time, professional training was provided to members of the group to enhance the intervention skills of the nursing staff, so that they could face complications such as bloodstream infections more calmly and give the child some emergency interventions to reduce the impact of complications on their clinical outcomes. Finally, an information-based intervention model and an information-based nursing quality assessment model were developed based on the work of the PICC room in the outpatient clinic.

We then implement an informational intervention model and introduce information systems: (1) firstly, information systems needed to be introduced to facilitate the implementation of an informational intervention model and informational quality of care assessment. Common information systems include hospital electronic medical record systems as well as QQ and WeChat platforms. (2) Secondly, information-based interventions could be implemented, i.e., when a child is admitted to a hospital, he or she can register online using the hospital's official website, WeChat public number, and other platforms and at the same time fill in basic information online on his or her own, and the system will create an electronic medical record file based on the patient's name and gender on its own. (3) When a child was seen, the physician would need to make detailed inquiries about his or her basic information, including checking his or her name and gender and taking a detailed record of the child's medical history and allergy history, etc. He or she will assess the child's specific condition based on his or her electronic medical record before prescribing tests. (4) PICC placement treatment based on the information system was positioned and fixed by the digital ultrasound machine, the relevant treatment was recorded in detail in the electronic medical record, and the first page of the medical record is maintained, including the position of positioning and puncture situation. After PICC placement, the nursing staff would ask the child's parents for contact details, including telephone number and address, and direct the child's family to join the PICC placement QQ group or WeChat group. The nursing staff should regularly send texts, pictures, and video screens related to health knowledge of PICC placement therapy to enhance the knowledge of PICC placement therapy and the self-care ability of the child and family members so that they are aware of the daily precautions after PICC placement. The nursing staff should be patient in answering questions or informing them of solutions that can be implemented. The child is followed up every 7 days in the clinic, and one-to-one online interventions are available to enquire about changes in the patient's condition and the catheter. After 3 months of PICC placement, the nursing staff could instruct the child and family to carry out a questionnaire on compliance, complications, and satisfaction to assess the child's treatment with the IT-based nursing intervention.

We evaluated the quality of information-based nursing: nursing staff can report on the meeting of the information-based nursing quality assessment group on a monthly, quarterly, and semiannual basis to discuss and analyze the diagnosis, treatment, and intervention of children with PICC at various stages and analyze relevant information based on electronic information, such as electronic medical records and group chat records. We counted the problems existing in the current nursing intervention and formulate improvement measures on time to continuously improve the daily work quality of the outpatient PICC room.

### 2.3. Observation Indicator

(1) The PICC placement maintenance status of the two groups of patients was statistically analyzed, including the PICC health knowledge score, compliance score, and the average time the catheter could be left in place. Patients' health knowledge was assessed using our own PICC health knowledge questionnaire, with a total score of 100; the higher the score, the better the knowledge of the child and/or family. A questionnaire was developed using the Delphi expert consultation method [4] to assess compliance with PICC placement in four areas: daily living habits, functional exercise, placement maintenance, and observation content. (2) The number of patients who developed catheter infection, catheter blockage or dislodgement, and peripheral phlebitis after the interventions were counted to compare which intervention helped the children to maintain a good and stable treatment status. (3) After the intervention, the child was able to maintain a good and stable status of PICC placement without complications such as catheter dislodgement and was able to grasp a more systematic and comprehensive knowledge of PICC health and was basically able to fully cooperate with the health care staff to complete the treatment and intervention. Satisfactory: after the intervention, the child's status of PICC placement was relatively stable, and no complications such as catheter dislodgement occurred, but the child fails to master systematic and comprehensive PICC health knowledge or sometimes does not cooperate with the health care personnel to complete the treatment and intervention and has resistance during part of the treatment stage. Unsatisfactory: after the intervention, if the child fails to maintain a good and stable PICC placement status, serious complications such as catheter dislodgement occur, and fails to master systematic and comprehensive PICC health knowledge with poor compliance during the consultation period. Overall satisfaction rate = (very satisfied + satisfied)/number of cases ∗ 100%.

### 2.4. Statistical Analysis

Statistical Product and Service Solutions (SPSS) 24.0 software (IBM, Armonk, NY, USA) was used to analyze the data information. *t*-test was used for measurement data, expressed as mean ± standard deviation, and *χ*^2^ test was used for count data, expressed as %. *P* < 0.05 was statistically significant.

## 3. Results

### 3.1. Comparison of Diagnosis and Treatment of PICC after Intervention between the Two Groups

After the intervention, compared with the control group, the PICC health knowledge mastery score, compliance score, and average catheter indwelling time of the children and/or their families were significantly higher in the observation group. The data comparison was statistically different (*P* < 0.05), as shown in Table 2.

### 3.2. Comparison of Complications after Intervention between the Two Groups

After intervention, the total incidence rate of complications in the observation group was lower than that in the control group. The data comparison was statistically different (*P* < 0.05), as shown in Table 3.

### 3.3. Comparison of Intervention Satisfaction between the Two Groups

After intervention, compared with the control group, the overall satisfaction rate of the children was significantly higher in the observation group. The data comparison was statistically significant (*P* < 0.05), as shown in Table 4.

## 4. Discussion

PICC is a more common clinical diagnosis and treatment, and generally, this diagnosis and treatment is mostly suitable for those who require long-term intravenous infusion therapy, those who require a repeated infusion of irritating drugs such as chemotherapeutic drugs, those who require a repeated infusion of blood products, those who require multiple venous blood draws for examination, those who require a long-term infusion of highly permeable or viscous drugs, or those who require infusion pumps [5]. Through PICC, it can not only reduce the pain caused by a repeated punctures to patients but also quickly disperse the drug to the whole body of patients while reducing the stimulation of related drugs to blood vessels, to achieve better drug diagnosis and treatment effect [6, 7].

However, as far as the clinical diagnosis and treatment of PICC are concerned, if the patients do not do a good job of self-protection during the diagnosis and treatment, if the arm activity range is too large or if the activity is too severe after catheterization, it is easy to cause complications such as catheter detachment, which will affect its diagnosis and treatment effect and diagnosis and treatment process. Therefore, to reduce the incidence of complications such as catheter detachment and improve the effect of PICC diagnosis and treatment for patients, this study intends to use the information nursing quality evaluation model to intervene in PICC patients to improve the quality of daily work in the outpatient PICC room. In this study, through the comparison of the information nursing quality evaluation model before and after the intervention, it can be seen that the PICC health knowledge mastery score of the observation group was 87.03 ± 8.43 (points), the compliance score was 53.77 ± 6.19 (points), and the average catheter indwelling time was 158.43 ± 28.32 (d); these three indicators of the control group were 80.01 ± 6.12 (points), 40.83 ± 5.98 (points), and 122.94 ± 25.98 (d), respectively, that is, the PICC health knowledge mastery score, compliance score, and average catheter indwelling time of the patients in the observation group after intervention. This is mainly due to the introduction of an information system in this intervention model, that is, through the establishment of electronic medical records, QQ group, microphone group, and the digitization of each patient's information through such as a platform, the nursing staff can obtain the patient's electronic medical record at any time and record the specific diagnosis and treatment of the patient at each diagnosis and treatment stage, PICC, etc. [8, 9]. At the same time, the PICC health knowledge will be pushed in the group regularly, so that the patients and their families have a deeper understanding of the relevant health knowledge and improve the patients' mastery of each health knowledge, so that the patients can know the necessity and importance of the relevant intervention measures so that they can more actively carry out PICC nursing and effectively improve their compliance in the diagnosis and treatment process [10, 11].

In terms of complications, the total incidence rate of complications was 1.51% in the observation group and 9.5% in the control group, that is, the total incidence rate of complications after the intervention was lower in the observation group. This is mainly because of patients can improve their self-care skills while receiving health education, and nursing staff can also answer questions for patients online, that is, once the patient's PICC is abnormal, nursing staff can timely guide patients online to implement certain intervention measures to reduce the incidence of complications such as catheter detachment [12, 13]. At the same time, with the in-depth understanding of relevant health knowledge by patients and their families, patients and their families can also have a deep understanding of the necessity and importance of each intervention measure, and the improvement of their compliance can enable patients to more cooperate with medical staff to complete various diagnosis, treatment, and intervention, which can reduce the incidence of complications such as catheter infection, avoid patients affecting the diagnosis and treatment process due to complications, and also avoid repeated puncture and other problems due to complications.

In terms of intervention satisfaction, the overall satisfaction rate of patients in the observation group was 98.87%; the overall satisfaction rate of the control group was 97.5%, i.e., the overall satisfaction rate of the observation group was higher. This is mainly because, in addition to the purely informational nursing intervention, the nursing staff will also conduct regular nursing quality assessments to summarize the nursing problems that exist at each stage and refer to the relevant informational and digital case information to develop more targeted interventions so that the patients can maintain a better and more stable PICC treatment state and enable them to achieve better clinical outcomes [14, 15]. The focus of this intervention model is that the nursing staff will not only provide information-based intervention care to patients but will also regularly discuss and summaries nursing problems and make reasonable use of modern information technology to summaries the nursing problems during the treatment of each PICC placement patient more conveniently through digital data and at the same time develop targeted interventions based on relevant index data to further optimize the quality of daily work in the outpatient. The quality of daily work in the PICC room is constantly being optimized and improved. This paper is a single-center randomized controlled study. The sample size is small, and the conclusions still need to be evaluated and verified by multicenter, large-scale, randomized clinical studies.

## 5. Conclusions

In conclusion, the information-based nursing quality assessment model can improve the quality of daily work in outpatient PICC rooms, enhance the clinical efficacy of PICC for patients, and reduce the incidence of complications such as catheter dislodgement and is worthy of clinical promotion and application.

## Figures and Tables

**Table 1:** Comparison of age and gender composition in the control group (*x̅* ± *s*, *n*).

Group	Number of subjects	Age range (months)	Mean age	Gender composition	
				Male	Female
Observation group	265	2–180	9.43 ± 2.11	161 (60.75%)	104 (39.25%)
Control group	200	3–168	9.48 ± 2.03	117 (58.5%)	83 (41.5%)
Χ^2^/*t*	—	—	0.257	0.241	0.241
*P*	—	—	0.797	0.623	0.623

**Table 2:** Comparison of diagnosis and treatment of PICC after intervention in the control group (*x̅* ± *s*).

Group	Number of subjects	PICC health knowledge score (points)	Compliance score (points)	Mean catheter dwell time (d)
Observation group	265	87.03 ± 8.43	53.77 ± 6.19	158.43 ± 28.32

Control group	200	80.01 ± 6.12	40.83 ± 5.98	122.94 ± 25.98
*t*	—	9.960	22.645	13.859
*P*	—	0.001	0.001	1.1

**Table 3:** Comparison of complications after intervention in control group (*n*, (%)).

Group	Number of subjects	Catheter infection	Catheter jams or falls off	Phlebitis peripheral	Total occurrence
Observation group	265	1 (0.38%)	2 (0.75%)	1 (0.38%)	4 (1.51%)
Control group	200	4 (2%)	8 (4%)	7 (3.5%)	19 (9.5%)
Χ^2^	—	2.821	5.705	6.573	15.479
*P*	—	0.093	0.017	0.010	1.1

**Table 4:** Comparison of intervention satisfaction rate in control group (*n*, (%)).

Group	Number of subjects	Very satisfied	Satisfied	Unsatisfactory	Overall satisfaction rate
Observation group	265	132 (49.81%)	130 (49.06%)	3 (1.13%)	232 (98.87%)
Control group	200	94 (47%)	101 (50.5%)	5 (2.5%)	195 (97.5%)
Χ^2^	—	0.361	0.095	1.261	15.046
*P*	—	0.548	0.758	0.261	0.001

## Data Availability

The datasets used and analyzed during the current study are available from the corresponding author on reasonable request.
